# Weighted Gene Coexpression Network Analysis Identified IL2/STAT5 Signaling Pathway as an Important Determinant of Peri-Implantitis

**DOI:** 10.1155/2022/4202823

**Published:** 2022-09-23

**Authors:** Li Tang, Hailun Zhou, Donghui Chen, Rong Xiang, Jianjia Tang

**Affiliations:** ^1^Department of Implant Dentistry, College of Stomatology, Guangxi Medical University, Nanning 530021, China; ^2^Guangxi Key Laboratory of the Rehabilitation and Reconstruction of Oral and Maxillofacial Research, Nanning 530021, China; ^3^Guangxi Colleges and Universities Key Laboratory of Treatment and Research for Oral and Maxillofacial Surgery Disease, Nanning 530021, China; ^4^Guangxi Clinical Research Center for Craniofacial Deformity, Nanning 530021, China

## Abstract

**Objective:**

Peri-implantitis (PI) is one of the main reasons for dental implant failure. Until now, the etiology and pathogenesis of PI remain unclear.

**Methods:**

In this study, we used differentially expressed genes (DEGs) analysis and gene function enrichment analysis to assess the expression profile of peri-implant bone tissue and gingiva in PI public data from the Gene Expression Omnibus (GEO) database. Then, we used gingival tissues from patients with PI and healthy individual to construct gene coexpression networks to reveal the biological functions of the genes in PI using RNA sequencing data. Afterward, key gene modules were selected to reveal the critical biological process or signaling pathway using Hallmark's gene enrichment and expression analysis of the related pathway members in PI.

**Results:**

DEGs were enriched in the formation of cellular responses to external stimuli in bone tissue. Cytokine production, lymphocyte activation, immune response-regulating signaling pathway, and blood vessel development were the top GO biology process or pathways of the DEGs in gingival tissue. Weighted gene coexpression network analysis (WGCNA) of RNA-seq data was used to assess the results of correlation analysis between modules and traits and correlation analysis between modules and functions. kMEpurple, kMEgreen, and kMEred modules were selected as the key gene modules. Signaling pathways and gene expression analysis were performed on selected modules, such as IL2/STAT5 signaling pathway, TNF*α* signaling pathway via NF*κ*B, and angiogenesis were enriched in kMEpurple module. Hedgehog signaling pathway, Wnt *β*-catenin signaling pathway, and IL2/STAT5 signaling pathway were enriched in kMEgreen module. Peroxisome, IL2/STAT5 signaling pathway, and epithelial-mesenchymal transformation process were enriched in kMEred module. All the enrichment results of key modules contained IL2/STAT5 signaling pathway*. Conclusion*. Differential gene and enrichment analysis based on public data showed differences in gene expression patterns and biological process between bone and gingival tissues in PI. This spatial-temporal heterogeneity is reflected in the formation of cellular responses to external stimuli, which was enriched in bone tissue, but cytokine production, lymphocyte activation, immune response regulating signaling pathway, and blood vessel development were enriched in gingival tissue. WGCNA and Hallmark gene sets enrichment analysis of the gingival tissue expression profile and showed that IL2-mediated activation of immune cells could be a critical mechanism in PI. As a new clinical treatment alternative, we suggest that IL2/STAT5 pathway blockers could be helpful in the treatment of PI.

## 1. Introduction

Dental implant, because of its advantages, such as perfect retention, less damage to adjacent teeth, and less foreign body sensation, has been widely used to reconstruct aesthetic and functional problems that result from teeth loss in clinic [1]. However, peri-implantitis (PI) characterized by infection of soft tissue and bone resorption is considered to be the result of an imbalance between the bacterial challenge, and the host response can affect the long-term success rate of dental implant, which is one of the main reasons for the failure of implant [2].

Bacterial invasion in the tissue surrounding implants can trigger an immune response. This response can remove harmful substances such as bacteria and toxins. However, the cytokines, proteases, and prostaglandins produced during this process can accelerate the destruction of tissue around the implants [3]. With the growing popularity of dental implants, PI has attracted considerable attention, but the etiology and pathogenesis are still unclear [4].

Weighted gene coexpression network analysis (WGCNA) [5] aims to find gene modules for coexpression and to explore the relationship between gene networks and phenotypes of interest, as well as the hub genes in the network. WGCNA could avoid the extensive false-positive and false-negative results of prior biological methods and exclude unreasonable statistical filtering in differential gene analysis. WGCNA has been widely used in cancer research, developmental biology, and systems biology [6, 7]. However, WGCNA is rarely used in the study of oral diseases.

In this study, we analyzed the expression profiles of peri-implant bone tissue and gingiva in PI from the GEO database using differentially expressed gene analysis and gene function enrichment analysis. Then, WGCNA was used to reveal the biological functions of the genes in PI. Owing to the similarity between genes and genes in the expression profiles data of probe-based PCR microarrays, the WGCNA of microarray data was failed to screen out gene modules and gene module members with biological significance. Therefore, we collected gingival tissues from patients with PI and healthy individual to construct gene coexpression network by RNA sequencing data. Next, we selected key modules to reveal the critical biological process or signaling pathway by Hallmark gene sets enrichment analysis and expression analysis of related pathways members in PI. In this study, we wish that high-throughput sequencing technology can be used to analyze the core issues that are plaguing the study of PI. Further, avoiding problems caused by defective technical means within basic medical research of peri-implantitis.

## 2. Material and Methods

### 2.1. Microarray Data Acquisition

Gene expression data were obtained from the Gene Expression Omnibus (GEO) database (https://www.ncbi.nlm.nih.gov/gds/). The datasets GSE57631 and GSE33774 were queried in the database using “peri-implantitis” as the search term. GSE57631contains 2 healthy peri-implantation bone tissues (BT_HI) and 6 peri-implantitis bone tissues (BT_PI) of expression profiling by array. GSE33774 contains 8 healthy peri-implantation gingival tissues (GT_HI) and 7 peri-implantitis gingival tissues (GT_PI) of expression profiling by array.

### 2.2. Microarray Data Analysis

*Z*-score was used to normalize the data. Then we used the differential genes analysis of expression matrix GEO2R (http://www.ncbi.nlm.nih.gov/geo/geo2r/). All the genes expression profiles were normalized using the R software package. Principal component analysis (PCA) and clustering analysis of expression patterns were performed using omicshare (http://www.omicshare.com).

### 2.3. Functional Enrichment Analysis of Microarray Data

Functional enrichment analysis was performed using the Metascape database (http://metascape.org/). KEGG pathway, GO biological processes, reactome gene sets, canonical pathways, and CORUM ontology were selected as sources. Terms with a *P* value <0.01, a minimum count of 3, and an enrichment factor > 1.5 were collected and grouped into clusters based on their similarities. Kappa scores were used as a metric of similarity when performing hierarchical clustering on the enriched terms, and sub-trees with a similarity of >0.3 were considered a cluster. The most statistically significant term within a cluster was chosen to represent the cluster. All the visualizations were performed using R software.

### 2.4. Weighted Gene Coexpression Network Analysis of Microarray Data

WGCNA is an algorithm used in gene coexpression network identification in profiles with different traits. In this section, R software package WGCNA was used to construct weighted coexpression networks to find key gene modules of interested within different traits.

### 2.5. Sample Collection

Gingival tissue samples of PI and healthy individual admitted to the Affiliated Stomatological Hospital of Guangxi Medical University were collected from December 2017 to December 2018. Inclusion criteria of gingival samples were described in the consensus report of the workgroup 4 in the 2017 World Workshop on the Classification of Periodontal and Peri-Implant Diseases and Conditions [2].

To obtain PI samples, the inflamed soft tissues around the implants were removed during an open surgical debridement following currently approved protocols. Gingival tissues from patients without any clinical infection were used a control. Control patients were operated due to wisdom teeth removals or teeth needed to be removed for orthodontics.

All the patients aged 18 years and above who did not smoke or drink alcohol were included, while we excluded patients with systemic diseases and other oral diseases, such as common mucous membrane disease, jaw cyst, and tumors. This study has been reviewed and approved by the Ethics Committee of Guangxi Medical University (2017-No. 165). All the patients agreed to participate in the study and signed informed consent before surgical intervention.

### 2.6. RNA Sequencing

Gingival tissue gene expression profiling was performed using RNA sequencing. Library construction was performed following the manufacturer's instructions provided by Illumina (San Diego, CA, USA). Samples were sequenced on an Illumina HiSeq 2500 instrument.

### 2.7. Weighted Gene Coexpression Network Analysis and Functional Enrichment Analysis of RNA-Seq Data

Same as WGCNA microarray data. The number of genes arranged in the constructed modules and functional enrichment analysis was performed on genes in these modules. The corresponding genes' information was mapped to Metascape (http://metascape.org/).

Hallmark gene sets were used as gene annotation source. Since the construction of the Molecular Signatures Database (MSigDB), it has been widely used as biological processes and diseases databases in metabolic disease and cancer. However, the increasing heterogeneity within gene sets is harmful to the utility of the database. Concerned with this situation, the hallmark gene sets were created as a part of MSigDB [8]. Each hallmark conveys a specific biological process and displays a coherent expression, which provides refined inputs for gene enrichment analysis. *P* value ≤0.05 after the correction was used as a threshold. The modules of interest were visualized using R software.

### 2.8. Statistics

The GraphPad Prism (Prism 8 for Windows, GraphPad Software Inc., San Diego, CA, USA) software was used for statistical analysis. Data obtained from the experiments are reported as the mean ± standard deviation (SD). The difference between the two groups was determined using Student's *t*-test. A *P* value of less than 0.05 was considered statistically significant.

## 3. Results

### 3.1. Differential Expression Gene Analysis from Microarray Data

We analyzed the expression profiles of genes in 2 healthy peri-implant bone tissue samples, 6 peri-implantitis bone tissues samples, 8 healthy gingival tissue samples, and 7 peri-implantitis gingival tissues samples. The results showed that 930 upregulated mRNAs and 1189 downregulated genes were identified in BT_HI-vs-BT_PI. Then 1735 significantly upregulated genes and 715 downregulated mRNAs were identified in GT_HI-vs-GT_PI. The list of top 20 DEGs is showed in Table 1.

To test the quality of the two-trait sample groups within expression profiles, the principal component analysis was used, as showed in Figure 1(a). The results of PCA analysis showed that the healthy bone tissue expression profiles and PI bone tissue of patients' expression profiles could be well distinguished, but there was a significant overlap between PI gingival tissue and healthy gingival tissue.

The expression pattern clustering the two-trait sample groups were shown in Figure 1(b). Clustering analysis of the expression patterns of genes with significant differences can adequately find the common points of expression among different genes and infer the similarity of gene functions according to the similarity of expression patterns. According to the results of the clustering analysis of expression patterns, the expression trends of gene groups with similar expression patterns in each sample can be expressed by curves. The distance calculation algorithm was used, the sample was Spearman, the gene was Pearson, and the clustering method was Hcluster.

### 3.2. Functional Enrichment Analysis of DEGs from Microarray Data

To test the biological function of the identified genes, information from differentially expressed genes were applied to the enrichment analysis using Metascape. Reactome gene sets, canonical pathways, CORUM, gene ontology (GO), and Kyoto encyclopedia of genes and genomes (KEGG) were used to obtain comprehensive functional annotations from multiple gene repositories for enrichment analysis.

The top 10 GO terms and pathways with the lowest *P* value of each group were shown in Table 2, and the results of the two groups enrichment were shown in Figure 1(c). DEGs were enriched in the formation of cellular responses to external stimuli in bone tissue. Moreover, cytokine production, lymphocyte activation, immune response regulating signaling pathway, and blood vessel development were the top GO biology process or pathways of DEGs in gingival tissue. It is suggested that the differential biological processes involved in the expression of gingival tissue genes and bone tissue genes may be the mechanism of spatiotemporal heterogeneity in peri-implantitis.

### 3.3. Weighted Gene Coexpression Network Analysis of Microarray Data

The individual gene variance in each sample was calculated according to the normalization of the expression profile. The unsigned network was constructed, selecting genes with a standard deviation higher than 1.2. The expression profiles and traits data consisted of 23 samples, 18357 genes, and 4 traits. Cluster analysis of all the samples was shown in Figure 2(a).

To ensure that the network is unsigned, the soft threshold value *β* = 6 was chosen. The expression profiles were transformed into the adjacency matrix and later transformed into the topological matrix. Based on the topological overlap measure (TOM), we used the average-linkage hierarchical clustering method to cluster genes. According to the standard of a hybrid dynamic cut tree, the minimum number of bases for each gene network module was 30. After determining the gene module with a dynamic splicing method, we calculate the eigengenes of each module, then cluster the modules, merge the nearer modules into new modules, and set the height = 6.94e − 17. Only three modules were obtained, as shown in Figure 2(b), in which the grey module is unable to aggregate into the gene set of other modules.

The gene significance of the members of module blue and turquoise was shown in Figure 2(c). The scatter plot of module kME value and gene significance value shows that higher the core value, smaller the *P* value, and the module members are more representative of the module characteristics.

### 3.4. Weighted Gene Coexpression Network Analysis of RNA-Seq Data

To test the quality of RNA sequencing within expression profiles, the principal component analysis was used, as shown in Figure 3(a). The results of PCA analysis showed that healthy gingival tissue expression profiles and PI gingival tissue of patients' expression profiles could be well distinguished, compared with the microarray data. Cluster analysis of all the samples was shown in Figure 3(b), and the gene dendrogram with traits was shown in Figure 3(c). It could be seen that genes were allocated to 11 modules, which could be used for function and module correlation analysis. According to the eigengenes of each module, the correlation between these modules and each trait was calculated, as shown in Figure 3(d).

kME was used to evaluate the value of effective connectivity between hub genes and to identify module members. Selecting the kME > 0.7 as the members of the modules, also named hub genes, can represent better the expression trend of the entire module. To reveal the functional correlation with gene module members, all the modules hub members were representative members of the module for gene enrichment analysis; the results were shown in Figure 3(e) and Table 3. Considering the results of the correlation analysis between modules and traits, and correlation analysis between modules and functions, the kMEpurple, kMEgreen, and kMEred modules were selected as the key gene modules. The gene significance of the members of the three modules was shown in Figure 4(a).

### 3.5. Signaling Pathway Analysis and Gene Expression Analysis of Key Gene Modules

The Hallmark gene sets were used as a source to reveal the critical biological process or signaling pathway of key gene modules using gene enrichment analysis. As shown in Figure 4(b), IL2/STAT5 signaling pathway, TNF*α* signaling pathway via NF*κ*B, and angiogenesis were enriched in kMEpurple module. Hedgehog signaling pathway, Wnt *β*-catenin signaling pathway, and IL2/STAT5 signaling pathway were enriched in kMEgreen module. Peroxisome, IL2/STAT5 signaling pathway, and epithelial-mesenchymal transformation process were enriched in kMEred module. All the enrichment results of key modules contained IL2/STAT5 signaling pathway. It is suggested that IL2-mediated activation of immune cells could be a critical mechanism in PI.

The gene expression of all the pathway members in different modules was plotted in Figure 5. The expression of some genes was inconsistent in bone and gingival tissues. More gene expressions were inconsistent in microarray and RNA sequencing data. These results confirm once again that difference in the expression of gingival tissue genes and bone tissue genes could be the mechanism of spatiotemporal heterogeneity in PI. The accuracy of gene expression profiles detected with microarray is inconsistent with RNA sequencing-based on next-generation sequencing.

## 4. Discussion

The development of molecular biology and bioinformatics has revolutionized pathology. Diseases are no longer considered to be caused by abnormal expression or single genes structural changes. Dynamic network relationships between genes and multiple negative feedbacks of signal pathways are considered important regulatory models of homeostasis against pathological factors [9]. To analyze the dynamic changes of gene expression profiles, weighted gene coexpression regulation analysis was created to explore the relationship between gene networks and phenotypes. It includes three steps: calculation of correlation coefficient between genes, constructed coexpression network, and determination of gene module with traits and function [5]. In this study, we firstly used WGCNA to reveal the PI mechanism and then identified IL2/STAT5 signaling pathway as a critical element in three key modules.

Previous studies demonstrated that the expression of cytokines stimulated by exogenous factors, degradation of the extracellular matrix [10], and cellular oxidative stress [11] is PI basic biological processes. This study confirmed these conclusions through the analysis of public databases. Moreover, through the comprehensive analysis of expression profiles, we found differences in gene expression patterns between bone and gingival tissues in PI. The differential genes of bone tissue were related to vascular growth and protein translation, processing, and transportation, while the differential genes in gingival tissues are involved in immune stress response. These differences in biological processes and cellular behavior expose the role of spatiotemporal heterogeneity in PI development. Previous studies have not considered the effects of different tissue behavior on disease occurrence. The gingival tissue is the first barrier against exogenous stimulants such as food debris, dental plaque [12], and implant dissolution [13]. It also plays a pioneering role in local tissue inflammation induced by host stress. Moreover, fibroblasts have been identified to be involved in PI pathogenesis by enhancing vascular and matrix degradation [14]. In clinical practice, uncontrolled PI has a poor prognosis leading to bone resorption, implant loosening, or loss. The proliferation of osteoclasts and apoptosis of osteoblasts is the cellular behaviors leading to this outcome. At the molecular level, active protein translation, processing, modification, and transport are the factors needed to complete this process.

The results of functional module gene enrichment analysis showed that IL2/STAT5 signaling pathway, TNF*α* signaling pathway via NF*κ*B, and angiogenesis were enriched in kMEpurple module. Hedgehog signaling pathway, Wnt *β*-catenin signaling pathway, and IL2/STAT5 signaling pathway were enriched in kMEgreen module. Peroxisome, IL2/STAT5 signaling pathway, and epithelial-mesenchymal transformation process were enriched in kMEred module. All the enrichment results of key modules contain IL2/STAT5 signaling pathway, has been suggested that IL2-mediated activation of immune cells play a critical mechanism in PI. IL2 receptor-dependent nuclear transcription factor STAT5 plays a key role in activating T_reg_ cells, and T_reg_ cells negatively regulate the body's immune response in vivo [15]. They usually play an important role in maintaining self-tolerance and avoiding body-injury by the immune response, but they also participate in immune surveillance and chronic infection [16, 17]. As an important pathway of host stress, the activation of Treg cells mediated by IL2/STAT5 signaling pathway is activated in PI gingival tissue. To some extent, this blocked the cascade amplification of inflammation signal and alleviated local tissue necrosis caused by inflammation and infection. However, this response is also an important way to induce host immune tolerance, causing persistent infection, and repeated clinical conditions [18]. This provides us with some clinical implications: IL2/STAT5 pathway blockers such as CMD178 [19] or pimozide [20] could be helpful in the PI treatment and inhibit T_reg_ cell activation at the pathway and molecular level.

In summary, there were differences in gene expression patterns and enriched biological process between bone and gingival tissues in PI, which means that biological processes and cellular behavior reveal the spatiotemporal heterogeneity in PI development. WGCNA and Hallmark gene enrichment analysis of the gingival tissue expression profile showed that IL2-mediated activation of immune cells could be a critical PI mechanism. As a new clinical treatment alternative, it is suggested that IL2/STAT5 pathway blockers could be helpful in PI treatment.

## 5. Conclusion

Differential gene and enrichment analysis based on public data showed differences in gene expression patterns and biological process between bone and gingival tissues in PI. This spatial-temporal heterogeneity is reflected in the formation of cellular responses to the external stimuli, which was enriched in bone tissue. In contrast, cytokine production, lymphocyte activation, immune response regulating signaling pathway, and blood vessel development were enriched in gingival tissue. WGCNA and Hallmark gene enrichment analysis of the gingival tissue expression profile showed that IL2-mediated activation of immune cells could be a critical PI mechanism. As a new clinical treatment, it is suggested that IL2/STAT5 pathway blockers could be helpful in PI treatment.

## Figures and Tables

**Figure 1:** Visualization of differentially expressed gene and enrichment analysis. (a) Principal component analysis of microarray expression profiles of bone and gingival tissue. (b) Cluster analysis of microarray expression profiles of bone and gingival tissue. (c) Heatmap of enriched terms across the differentially expressed gene, colored by *P* values.

**Figure 2:** Weighted gene coexpression network analysis of microarray data. (a) Sample dendrogram and trait heatmap: the red representation in the graph is marked as nonzero samples in the trait data. (b) Gene dendrogram with trait: this figure is divided into three parts. The first part is the phylogenetic clustering tree of genes. The second part shows the module color display of the corresponding genes. The third part shows the correlation between the genes in each character-related sample and its module. The redder the color, the more positive the correlation. The negative correlation is blue. (c) Gene saliency map of module blue and turquoise members: scatter plot of module kME value and gene saliency value, higher the core value, smaller the *P* value, and the module members can represent the module characteristics better.

**Figure 3:** Weighted Gene coexpression network analysis of RNA-seq data. (a) Principal component analysis of RNA-seq expression profiles of gingival tissue. (b) Sample dendrogram and trait heatmap of RNA-seq data. (c) Gene dendrogram with a trait of RNA-seq data. (d) Module-trait correlation thermograms: correlation of thermograms between modules and given traits. The closer the correlation between trait and module to the absolute value of 1; the trait is related to the gene function of the module. (e) Heatmap of enriched terms across module gene members, colored by *P* values.

**Figure 4:** Significance analysis and signaling pathway analysis of key gene Modules. (a) Gene saliency map of module purple, green, and red members. (b) Column graphs of enriched terms across three modules genes members, colored by *P* values.

**Figure 5:** Genes expression analysis of key gene modules. Expression of key gene module members.

**Table 1:** List of top 20 differentially expressed genes.

Gene	Description	logFC	*P* value	FDR
BT_HI-vs-BT_PI				
ZMPSTE24	Zinc metallopeptidase STE24	0.05436861	0.000425	0.418
TUBB4B	Tubulin beta 4B class IVb	0.067058028	0.000776	0.418
EIF3M	Eukaryotic translation initiation factor 3 subunit M	0.163804868	0.000305	0.418
RAB10	RAB10, member RAS oncogene family	0.144274808	0.000823	0.418
SF3A3	Splicing factor 3a subunit 3	0.040577086	0.001089	0.418
AP1G1	Adaptor related prot	0.056817586	0.001125	0.418
C20orf203	Chromosome 20 open reading frame 203	-0.129391728	0.000552	0.418
MIR15B	microRNA 15b	-0.141409803	0.000692	0.418
MIR214	microRNA 214	-0.115661557	0.000828	0.418
MIR99A	microRNA 99a	-0.073109217	0.001108	0.418
OCIAD1	OCIA domain containing 1	0.123431672	0.001013	0.418
CAV1	Caveolin 1	0.093133672	0.00071	0.418
BRK1	BRICK1 subunit of SCAR/WAVE actin nucleating complex	0.065658554	0.000527	0.418
PPP6C	Protein phosphatase 6 catalytic subunit	0.03378179	0.000684	0.418
PSMB3	Proteasome subunit beta 3	0.135521691	0.000908	0.418
PSMD10	Proteasome 26S subunit, non-ATPase 10	-0.152847334	0.000283	0.418
HIST1H2BG	Histone cluster 1 H2B family member g	0.112335029	0.000385	0.418
SNRPG	Small nuclear ribonucleoprotein polypeptide G	0.149342222	0.000241	0.418
DCTN5	Dynactin subunit 5	0.119709276	0.000526	0.418
CAPZA1	Capping actin protein of muscle Z-line subunit alpha 1	0.145481101	0.000343	0.418
GT_HI-vs-GT_PI				
NEFM	Neurofilament, medium polypeptide	-1.4062788	0.00000032	0.0106
MAPT	Microtubule associated protein tau	-1.83338262	0.00000206	0.0246
MERTK	MER proto-oncogene, tyrosine kinase	1.01973984	0.00000295	0.0246
MRC1	Mannose receptor, C type 1	1.01068439	0.00000588	0.029
GLIPR2	GLI pathogenesis related 2	0.86823054	0.00000688	0.029
SLC2A3	Solute carrier family 2 member 3	1.26464786	0.00000736	0.029
SLCO2B1	Solute carrier organic anion transporter family member 2B1	0.84589762	0.00000911	0.029
SRPX2	Sushi repeat containing protein, *X*-linked 2	1.27391664	0.00000938	0.029
CD14	CD14 molecule	1.33965561	0.00000996	0.029
MSR1	Macrophage scavenger receptor 1	1.17709016	0.00001044	0.029
C1QB	Complement C1q B chain	0.83761875	0.00001224	0.0313
STAC2	SH3 and cysteine rich domain 2	-1.18651859	0.00001325	0.0313
CHRNA3	Cholinergic receptor nicotinic alpha 3 subunit	-0.94702121	0.00001433	0.0313
CTGF	Connective tissue growth factor	1.32968345	0.00001505	0.0313
CASP10	Caspase 10	0.66524239	0.00001683	0.033
TLR4	Toll like receptor 4	1.40463223	0.00001948	0.036
MS4A6A	Membrane spanning 4-domains A6A	0.91872666	0.00002886	0.0494
C3AR1	Complement component 3a receptor 1	1.07948921	0.00003202	0.0494
CMAHP	Cytidine monophospho-N-acetylneuraminic acid hydroxylase, pseudogene	0.79185305	0.00003378	0.0494
SRGN	Serglycin	1.37684391	0.00003424	0.0494

**Table 2:** List of top 10 enriched GO terms and pathways.

GO	Category	Description	Count	%	Log10 (*P*)	Log10 (*q*)
BT_HI-vs-BT_PI						
R-HSA-8953897	Reactome gene sets	Cellular responses to external stimuli	105	5.1	-15.97	-11.66
hsa04141	KEGG pathway	Protein processing in endoplasmic reticulum	46	2.23	-12.45	-9.03
GO:0006888	GO biological processes	ER to Golgi vesicle-mediated transport	54	2.62	-12.3	-8.94
R-HSA-6798695	Reactome gene sets	Neutrophil degranulation	86	4.18	-10.54	-7.42
R-HSA-5619115	Reactome gene sets	Disorders of transmembrane transporters	43	2.09	-9.82	-6.99
GO:0048514	GO biological processes	Blood vessel morphogenesis	105	5.1	-8.45	-5.95
GO:0006412	GO biological processes	Translation	108	5.25	-8.39	-5.91
GO:0044257	GO biological processes	Cellular protein catabolic process	110	5.34	-7.33	-5.06
R-HSA-72766	Reactome gene sets	Translation	52	2.53	-6.6	-4.44
GO:0060627	GO biological processes	Regulation of vesicle-mediated transport	81	3.93	-6.57	-4.42
GT_HI-vs-GT_PI						
GO:0002274	GO biological processes	Myeloid leukocyte activation	194	8.1	-45.73	-41.42
GO:0046649	GO biological processes	Lymphocyte activation	200	8.35	-40.59	-36.88
GO:0040017	GO biological processes	Positive regulation of locomotion	162	6.76	-33.22	-29.8
GO:0050900	GO biological processes	Leukocyte migration	143	5.97	-31.7	-28.56
GO:0001568	GO biological processes	Blood vessel development	183	7.64	-29.38	-26.44
GO:0043062	GO biological processes	Extracellular structure organization	124	5.18	-28.7	-25.81
GO:0001816	GO biological processes	Cytokine production	179	7.47	-25.89	-23.11
R-HSA-109582	Reactome gene sets	Hemostasis	147	6.14	-23.42	-20.68
GO:0002764	GO biological processes	Immune response-regulating signaling pathway	153	6.39	-22.13	-19.41
GO:0030029	GO biological processes	Actin filament-based process	164	6.84	-21.6	-18.9

**Table 3:** Enrichment analysis results of modules.

Module	GO	Description	Log10 (*P*)
kMEblack	GO:0002250	Adaptive immune response	-7.69
	GO:0042113	B cell activation	-6.40
	GO:0097190	Apoptotic signaling pathway	-6.12
	GO:0002285	Lymphocyte activation involved in immune response	-4.83
	GO:0001816	Cytokine production	-4.63
kMEblue	GO:0001816	Cytokine production	-35.63
	GO:0030155	Regulation of cell adhesion	-33.09
	GO:0002250	Adaptive immune response	-32.10
	GO:0002366	Leukocyte activation involved in immune response	-28.75
	GO:0019221	Cytokine-mediated signaling pathway	-26.74
kMEcyan	GO:0002366	Leukocyte activation involved in immune response	-14.65
	GO:0019221	Cytokine-mediated signaling pathway	-14.53
	hsa04060	Cytokine-cytokine receptor interaction	-13.45
	GO:0042330	Taxis	-11.47
	GO:0009617	Response to bacterium	-10.84
kMEdarkred	R-HSA-6809371	Formation of the cornified envelope	-6.80
	GO:0042552	Myelination	-3.54
	GO:0008203	Cholesterol metabolic process	-3.36
	GO:0016485	Protein processing	-2.38
	M5885	NABA matrisome associated	-2.22
kMEgreen	GO:0008544	Epidermis development	-26.58
	GO:0001942	Hair follicle development	-12.11
	GO:0048729	Tissue morphogenesis	-9.51
	GO:0008610	Lipid biosynthetic process	-6.79
	GO:0000904	Cell morphogenesis involved in differentiation	-6.75
kMElightcyan	GO:0042113	B cell activation	-10.34
	GO:0002366	Leukocyte activation involved in immune response	-8.24
	GO:0002253	Activation of immune response	-8.06
	R-HSA-1280218	Adaptive immune system	-7.80
	GO:0002250	Adaptive immune response	-7.76
kMElightgreen	GO:0070268	Cornification	-13.86
	GO:0008544	Epidermis development	-11.51
	GO:0070841	Inclusion body assembly	-6.97
	R-HSA-1461957	Beta defensins	-4.12
	GO:0033559	Unsaturated fatty acid metabolic process	-2.86
kMEmidnightblue	GO:0009617	Response to bacterium	-7.61
	GO:0002366	Leukocyte activation involved in immune response	-7.51
	hsa05150	Staphylococcus aureus infection	-6.94
	GO:0007249	I-kappaB kinase/NF-kappaB signaling	-6.77
	GO:0001816	Cytokine production	-6.55
kMEpurple	GO:0000904	Cell morphogenesis involved in differentiation	-4.37
	GO:0048729	Tissue morphogenesis	-3.87
	GO:0048598	Embryonic morphogenesis	-3.62
	GO:0022604	Regulation of cell morphogenesis	-3.52
	GO:0030155	Regulation of cell adhesion	-3.29
kMEred	R-HSA-156902	Peptide chain elongation	-7.09
	R-HSA-201681	TCF dependent signaling in response to WNT	-4.97
	GO:0033131	Regulation of glucokinase activity	-3.45
	GO:0051013	Microtubule severing	-3.32
	GO:0090277	Positive regulation of peptide hormone secretion	-3.28
kMEroyalblue	GO:0001503	Ossification	-4.32
	GO:0001501	Skeletal system development	-3.78
	hsa04514	Cell adhesion molecules (CAMs)	-3.35
	GO:0045596	Negative regulation of cell differentiation	-3.02
	GO:0010942	Positive regulation of cell death	-2.21

## Data Availability

The datasets used and analyzed during the current study are available from the corresponding author on reasonable request.
